# Remodeling of Lumbar Spinal Osteoid Osteoma Resected With Microscopic Surgery in a 15-Year-Old Basketball Player: A Case Report

**DOI:** 10.7759/cureus.48351

**Published:** 2023-11-06

**Authors:** Shogo Matsumoto, Ukei Anazawa, Aya Sasaki, Hiraku Hotta, Itsuo Watanabe, Ryoma Aoyama

**Affiliations:** 1 Orthopaedic Surgery, Tokyo Dental College Ichikawa General Hospital, Ichikawa, JPN; 2 Clinical Laboratory, Tokyo Dental College Ichikawa General Hospital, Ichikawa, JPN; 3 Rehabilitation, Tokyo Dental College Ichikawa General Hospital, Ichikawa, JPN

**Keywords:** youth sports, spine oncology, basketball player, microscopic surgery, remodeling, osteoid osteoma

## Abstract

This case report focuses on a 15-year-old competitive-level high school basketball player who experienced chronic low back pain. Diagnostic imaging revealed osteoid osteoma in the L5 posterior element, causing osteosclerotic deformity of the left lamina and more inferior facet. To return him to the condition of sports activity, less invasive surgery of microscopic tumor resection with autologous bone grafting was planned instead of CT-guided ablation, which can cause thermal injury to nearby tissues.

This procedure could preserve spinal structures, including the facet, pedicle, and paravertebral muscles. The day after surgery, the patient experienced a complete resolution of lower back pain. He gradually resumed light exercise two months postoperatively. Three-month follow-up CT imaging revealed bone remodeling at the resection site, to return to complete basketball activities. Over five years, no tumor recurrence or symptoms were observed, and he maintained his competitive activity level.

## Introduction

Osteoid osteoma (OO) is a benign bone tumor representing approximately 3% of all primary bone tumors [1]. This tumor is more common in the 10-30 years age group. Radiologically, it is characterized by nidus, a lesion surrounding the radiolucent zone with osteosclerosis, often resulting in bony deformity with bone hyperplasia on X-ray and CT images. The tumor also causes inflammatory changes around the lesion, which is radiologically revealed on MRI [2]. Clinically, it causes nocturnal pain that is relieved with nonsteroidal anti-inflammatory drugs (NSAIDs). OO occurring in the spine is rare and is one of the differential diagnoses of lower back pain in young patients [3], but it may take time to diagnose accurately. Treatment of OO is sufficient with only excision of the nidus, and percutaneous ablation has been famous as a minimally invasive surgery. However, ablation can result in a reactive change in the typical bone and muscle structures, and this bone degenerative change remains for over one year.

We report a case of a 15-year-old basketball player with chronic low back pain who presented with OO in the L5 posterior bone, and the tumor caused osteosclerotic deformity of the left lamina and more inferior facet. In this case, minimally invasive microscopic tumor resection with autologous bone grafting was performed, and bone remodeling at the resection site was confirmed three months after surgery, allowing the patient to return to complete basketball activities.

## Case presentation

A 15-year-old boy, a competitive-level high school basketball player, presented with a three-year history of persistent lower back pain. The pain had increased at night and on playing basketball. He played basketball while being treated with NSAIDs. Gradually, the pain increased and became painful during the day, even without playing sports. X-ray and magnetic resonance imaging (MRI) showed abnormalities in the left posterior spine and muscles at the L5 level, and he was referred to our clinic. Physical examination revealed only stiffness and tenderness in the left side of the lumbosacral region without neurological abnormality. Laboratory examinations demonstrated no apparent anomaly. The time to run 50 m was 7.19 seconds. X-ray showed spina bifida occulta in the L5 lamina with osteosclerotic deformities of the left lamina and inferior articular process (Figure 1).

**Figure 1:** A simple lumbar X-ray at the time of the initial examination. (A) Front view, (B) lateral view, and (C) oblique view. Slight scoliosis was shown, and spina bifida at L5 with osteosclerotic deformity of the right lamina and inferior articular process were confirmed (red arrow).

Computed tomography (CT) revealed a radiolucent lesion 18 mm long in diameter with multiple calcifications extending from the left lamina to the inferior articular process (Figure 2). The lesions were surrounded by sclerotic zones extending into the pedicle and showed hyperplastic deformities. MRI showed the lesion with intermediate signal intensity on T1- and T2-weighted images (WI). On T2WI, bone and soft tissue around the lesion, including paravertebral muscle, showed high signal intensities, suggesting inflammatory change (Figure 3).

**Figure 2:** Simple CT (A) sagittal, (B) axial, and (C) coronal images of the lumbar spine at the initial examination. A radiolucent lesion, nidus of 18 mm in diameter with multiple calcifications, was revealed in the left L5 inferior articular process. The sclerotic zone around the lesion extending into the pedicle was shown, and hyperplasia of the lamina and the inferior articular process was demonstrated.

**Figure 3:** T1- and T2-weighted sagittal images (A, B) and T2-weighted axial image (C) of MRI at the initial examination. The lesion was iso signal intense in both T1- and T2-weighted images (red arrow). The base of the pedicle and paravertebral muscle showed high signal intensities, suggesting inflammation change around the lesion.

This painful lesion was clinically and radiologically diagnosed as OO because it was a radiolucent lesion, nidus, surrounded by osteosclerotic deformity and associated with inflammatory changes.

Gradually, NSAIDs no longer controlled local pain, and this patient could not continue playing competition-level basketball. Therefore, tumor excision was indicated. To prevent unnecessary surgical invasion of bone and soft tissue and ensure early bone remodeling, microscopic tumor curettage with autologous bone grafting, expected to replace the normal bone structure, was performed with microscopic mini-open surgery. This procedure involved an incision approximately 1 cm from the midline, passing through the paravertebral muscles to directly reach the spinal posterior lesion. After exposing the tumor portion of the lamina to the inferior articular process, a microscopic view revealed abnormal roughening and hyperemia of the bone surface in this area. This abnormal bone cortex was excised with a high-speed burr, and a lesion that was gritty red-brown-colored tissue could be identified beneath it. The lesion was treated with curettage thoroughly, and the surrounding osteosclerotic area and normal bone marrow tissue were visualized. Then, autologous bone harvested from the posterior iliac crest was grafted into the bone defect after removing the tumor (Figure 4).

**Figure 4:** Intraoperative photograph. The bone surface of the lamina to the inferior articular process (red arrow) was roughening and hyperemia. A gritty and red-brown-colored lesion was identified beneath this abnormal bone cortex and excised with a small curette (A). Curettage was removed (B) until the area of osteosclerosis and normal bone marrow was recognized (C).

Histopathologic examination revealed the presence of immature bone and a highly vascularized osteoid, and pathologically, it was diagnosed as OO (Figure 5).

**Figure 5:** Histopathological image. Immature bone and osteoid bone-like tissue are observed, with surrounding vascular growth.

The lower back pain completely resolved the day after surgery. The patient was discharged with a lumbosacral corset and could perform activities of daily living. Two months later, he was allowed light exercise. Three months after surgery, CT imaging showed bone remodeling at the resection site (Figure 6), and he was allowed full exercise. Four months after surgery, the patient returned to basketball tournaments without problems. His performance improved from 7.19 seconds to 6.29 seconds in the 50 m run before and one year after surgery. Five years after surgery, there has been no tumor recurrence or symptoms.

**Figure 6:** CT images immediately postoperatively (A: axial; B: coronal) and three months postoperatively (C: axial; D: coronal). Bone remodeling of the lesion was observed at three months postoperatively (red arrow).

## Discussion

OO principally occurs in the long bones of the lower extremities, with tumors measuring less than 20 mm in size [4]. The tumor is radiographically characterized by nidus, a radiolucent zone of the tumor with surrounding reactive osteosclerosis, and clinically by nocturnal pain in response to NSAIDs and showed an inflammatory change in the tissues surrounding the lesion [5]. On MRI, inflammatory reactions centered on the tumor are often seen as high-signal areas on T2-weighted images [2]. OO occurring in the spine are rare, representing approximately 10% of them, and almost arise in the posterior element of the spine [6]. It usually presents with back pain that worsens at night and is relieved by NSAIDs. In the case of spinal OO occurring near nerve roots, lumbar herniation-like neuropathies could be caused, which may take a long time to diagnose.

This tumor could be treated with conservative or surgical treatment. Conservative therapy consists of the oral administration of NSAIDs and may require a more extended treatment period of one year or more. This administration could lead to side effects of NSAIDs. In addition, long-term pain and inflammatory conditions can lead to overgrowth or deformity of affected bones, such as spinal scoliosis [7]. Therefore, surgery is often considered for early healing in younger patients.

For surgical treatment, resection of the nidus only is sufficient. However, because the lesion is small and surrounded by osteosclerotic bone, it is difficult to identify the nidus grossly during surgery. Despite the small size of the lesion, resection of this tumor requires excessive surgical invasion of the bone and soft tissue around the nidus.

In recent years, CT-guided tumor resection and ablation have been more common for treating OO to minimize surgical invasion [5]. CT-guided percutaneous radiofrequency ablation has been performed due to its advantage of reducing damage to bone and soft tissues, and it has become the mainstay of treatment in cases of the extremities and pelvis [8]. This procedure can achieve remission of symptoms in 78-93% of the patients and does not damage the surrounding tissues [8,9] so that patients can return to their daily lives early after surgery. If symptoms remain, they can be treated again using the same CT-guiding technique. While radiofrequency ablation can cause thermal changes in the ablated area, it was reported that radiofrequency ablation could cause degenerative changes in bone tissue in a sphere of approximately 9-13 mm [10]. Vanderschueren et al. demonstrated imaging findings of this lesion after radiofrequency ablation and reported 63 patients with remission of symptoms. On CT images, one year after surgery, only seven (20%) showed complete bone formation of the ablated area, and the rest showed localized thermal necrosis or residual nidus. On MRI, normalization of edema-like reactive changes in the bone and soft tissue around the lesions was observed at only 23% one year after initial treatment [11]. These suggest that radiofrequency ablation may result in long-term pathological conditions of bony structures after surgery.

On surgical resection of spinal OO, Quraishi et al. reported 84 cases treated with en-bloc resection and curettage. They demonstrated that local recurrence occurred in 7% of patients with curettage alone and no repeat with en-bloc resection [12]. On the other hand, en-bloc resection may cause postoperative instability depending on the location and size of the tumor, requiring posterior fixation [13]. This suggested that en-bloc resection should be avoided, but it should be considered if the nidus can be completely removed with curettage. On the other hand, there are increasing reports of microscopic and endoscopic tumor resection techniques that are less invasive to the soft tissues surrounding the tumor and can allow for correct tumor resection without ablation therapy [14,15].

In our case, surgical treatment was performed because the goal of treatment was to allow the patient to play basketball. Since the lesion extends from the lamina to the inferior articular process and affects the intervertebral joints in the condition of spina bifida occulta, there was concern that CT-guided ablation could lead to local complications such as spondylolysis and suppression of remodeling due to thermal degeneration change. Therefore, microscopic curettage of the tumor was performed to minimize damage to the bone and soft tissue surrounding the lesion and to achieve complete resection, followed by autologous bone grafting at the resection site in anticipation of early bone remodeling.

Mini-open surgeries with endoscopic or microscopic techniques, which can preserve the intervertebral joints and the pedicle for OOs of the posterior spine, allow for a better surgical field of view and complete tumor resection [14-16]. Hikata et al. reported a case of cervical spinal OO treated with microendoscopic resection and demonstrated remodeling in the resected site at one year postoperative CT [17]. Kotheeranurak et al. presented a lumbar spinal OO treated with endoscopic resection, showing remodeling of the lumbar facet joint at two years postoperative CT [18]. These suggested that bone remodeling can be expected within one to two years after endoscopic and microscopic, less invasive surgery of the spinal OO.

In our case of lumbar OO in L5 lamina showing spina bifida occulta, a less invasive procedure of microscopic resection followed by autogenous bone graft, preserving posterior spinal structures including the facet, pedicle, and paravertebral muscles, could show the remodeling of bone defects at three months postoperative CT and allow the patient to resume playing basketball.

## Conclusions

Minimally invasive microscopic tumor resection with autologous bone grafting was performed on a basketball player, and bone remodeling at the resection site was confirmed three months after surgery, allowing the patient to return to complete basketball activities.
